RETRACTED

# Exploring Online Teaching Design of Curriculum Politics by Deep Learning and Visual Sensing Technology

**DOI:** 10.1155/2022/1283256

**Published:** 2022-05-04

**Authors:** XiaoJuan Huang, Yanhong Xie, Yongyu Li

**Affiliations:** ^1^College of Finance and Economics Management, Guangzhou Institute of Technology, Guangzhou 510075, Guangdong, China; ^2^Maxim Healthcare Service, Washington State, WA, USA

## Abstract

The study aims to explore the online teaching design of ideological and political education (IPE). Based on the relevant theories of deep learning (DL) and visual sensing, the students of a Chinese University are taken as the research samples and investigated by a questionnaire survey. Then, DL and visual sensing are introduced into the online teaching design of IPE, and the research conclusions are obtained. The results show that college students are interested in IPE, but there are still some problems in the actual teaching process. For example, 60% of the students do not know the learning objectives of IPE, and 19.7% are not familiar with the learning contents; based on the image semantic analysis of the curriculum of IPE, DL mainly focuses on model construction and data processing, and visual sensing is used to classify image pixels; the students' concentration time is changed from 29 minutes to 30.4 minutes, and their efficiency of homework submission is also improved based on DL and visual sensing. The study has a great reference for ideological and political teaching in the future.

## 1. Introduction

*The Seminar on Teachers of Ideological and Political Theory in School Curriculum* was held in March 2019. At the symposium, China's President Xi Jinping pointed out “it is necessary to set up theories for curriculum politics step by step and spirally in primary and secondary schools, which is an important guarantee for cultivating generations of socialist builders and successors [1].” The curriculum politics are politically important. There is an urgent need to consider how to make them more conducive to students' learning so that they can have a more in-depth and flexible understanding of them [2].

Zhu (2019) expounded that the curriculum politics were guided by the basic standpoint and method of Marxism. School courses should be regarded as the carrier of political education. The political education should be through the whole process of teaching links, to form an omnidirectional, multiangle, and three-dimensional curriculum system [3]. Shi (2018) concluded that the essence of curriculum politics was to cultivate students by virtue, whose concept was collaborative education and whose structure was three-dimensional and diversified. The method of curriculum politics is the combination of explicit and implicit knowledge, and its thinking result is scientific innovation [4]. Mandalorian (2018) believed that the transformation of the ideological and political curriculum into curriculum politics was conducive to the innovative development of school ideological and political education (IPE), changing the traditional IPE mode, optimizing and innovating the curriculum teaching content, and improving the effectiveness and applicability of IPE [5]. Saussure (2018) reckoned that professional teachers should improve their literacy and ability, deeply explore ideological and political elements in professional teaching, strengthen mutual assistance and cooperation with ideological and political teachers, and jointly realize collaborative education [6]. Tissters (2019) signified that the primary task of integrating DL and visual sensing technology into curriculum politics was to strengthen the theoretical research about curriculum politics, do a good job in top-level design, coordinate and promote ideological and political construction on students, and strengthen the construction of characteristic specialty groups [7].

RETRACTED

Based on the above, a questionnaire survey is designed to know college students' motivation and behavior in IPE. Then, the teaching design of IPE integrated with DL and visual sensing is analyzed. Although some great achievements have been made in the relevant fields, there is still some room to be improved. According to the theory and some experiments, the application of DL and visual sensing to the teaching design of IPE is analyzed. The main task is to analyze the role of DL and visual sensing in optimizing the online teaching design of IPE.

## 2. Materials and Methods

### 2.1. Analysis of Online Curriculum Politics Based on DL Model

The goal of curriculum politics is to build an all-around education pattern with the participation of all members in the society so that all courses and ideological and political courses can walk in the same direction and form a synergistic effect [8, 9]. From the macro level, the method of curriculum politics is to integrate different ideological and political elements with various professional courses and to realize the collaborative education in classroom teaching. From the microlevel, the concept of curriculum politics is a kind of curriculum view. It is not to set up a new curriculum in the school but to combine IPE with professional knowledge through a scientific teaching design in a specific curriculum. The content of the curriculum politics is mainly composed of four parts of theoretical basis [10].  Figure 1 demonstrates the theoretical basis of curriculum politics.

RETRACTED

DL is adopted to explore the internal law and representation level of data from the learning sample. The information obtained in the learning process is very helpful to the interpreting data such as text, image, and sound. Its goal is to enable the machine to have the same analyzing and learning ability as humans and to recognize data such as text, image, and sound [11]. DL is a new research direction in the field of machine learning (ML). Its operation principle is to use a neural network to realize the simulation of analysis and learning like the human brain. ML is a technology that studies how computers simulate or realize the learning behavior of animals, to learn new knowledge or skills, rewrite the existing data structure, and then improve the program performance. DL neural network is a technology in the field of ML. This technology simulates the human brain neuron structure by constructing a multilayer network, iteratively analyzes the data layer by layer, and continuously extracts features, to obtain the essential features of the initial data, which has a good effect on solving the classification problem. Compared with the traditional classification method, it greatly reduces the complexity in the extraction of features and data reconstruction [12].  Figure 2 illustrates its specific model.

The judgment basis of the DL algorithm is to correct the weight and deviation of the neuron layer by observing the decline degree of error function of the whole neural network. The following equation displays its calculation method:

(1) $$\begin{array}{c} Q_{a+1}=Q_{a}-c_{a}d_{a}. \end{array}$$

In equation (1), *Q*_*a*_ represents the weight and deviation value of the network, *Q*_*a*+1_ denotes the weight and deviation value after iterative calculation, *c*_*a*_ refers to the learning speed of the neural network, and *d*_*a*_ stands for the gradient of the error function.

The following equation indicates the propagation process algorithm of DL:

(2) $$\begin{array}{c} C_{0}=x. \end{array}$$

In equation (2), *x* is the model input, and *C*_0_ accords to the regular term coefficient.

(3) $$\begin{array}{c} P_{l}=W_{l}a_{l-1}+b_{l}. \end{array}$$

In equation (3), *P*_*l*_ denotes the input for each layer, *l* represents the network depth (*l* ∈ (1, *L*), and it is an integer), *W*_*l*_ refers to the weight matrix in the *l*th layer, and *b*_*l*_ stands for the offset vector in the *l*th layer. The meanings of the remaining letters are the same as equation (2).

(4) $$\begin{array}{c} b_{l}=f\left(P_{l}\right). \end{array}$$

In equation (4), the letters mean the same as in equation (3).

(5) $$\begin{array}{c} y^{\prime }=b_{E}. \end{array}$$

In equation (5), *y*′ expresses the network output value, and *b*_*E*_ means the output value of *E*th layer (the last layer).

(6) $$\begin{array}{c} H=L\left(y^{\prime },y\right)+b\delta \left(\vartheta \right). \end{array}$$

In equation (6), *H* stands for the loss function, *y* denotes the real value corresponding to the input sample, *L*(*y*′, *y*) represents the difference between the real value corresponding to the input sample and the network output value, and *δ*(*ϑ*) represents a regular term added to prevent overfitting of the model, including all parameters *W* and *b* in the model.

RETRACTED

DL is a general term for a class of pattern analysis methods, which mainly involves three types of methods: convolutional neural network (CNN), recurrent neural network (RNN), and generative adversarial network (GAN) [13].

(1) RNN is an artificial neural network (ANN) with a tree hierarchical structure, and the network nodes recur the input information according to its connection order. It is one of the DL algorithms [14, 15]. RNN has a changeable topology and weight sharing. They are used in machine learning tasks containing structural relationships. They attract much attention in natural language processing (NLP). The specific model is shown in Figure 3.
(2) CNN includes convolution calculation and calculates feedforward neural networks with a deep structure. It is mainly divided into four parts: the input layer, convolution layer, pooling layer, and fully connected layer. It is one of the representative algorithms of DL [16]. The model is shown in Figure 4.
The principle of the CNN model is to randomly select samples from the sample set as a training set and then give the target output vector to calculate the output error term. The following equation signifies the specific calculation method.
  (7) $$\begin{array}{c} \delta_{k}=\left(d_{k}-y_{k}\right)y_{k}\left(1-y_{k}\right). \end{array}$$
In equation (7), *δ*_*k*_ represents the output error term, *d*_*k*_ denotes the element in the target vector, and *y*_*k*_ refers to an element in the output vector.
The following equation manifests the calculation of the hidden element error term of the middle layer.
  (8) $$\begin{array}{c} \delta_{j}=h_{j}\left(1-h_{j}\right)\sum_{k=0}^{M-1}\delta_{k}W_{jk}. \end{array}$$
In equation (8), *δ*_*j*_ denotes the error term of the hidden element, *h*_*j*_ means the output vector of the middle layer, *M* bespeaks the sample, *k* expresses the element, and *W*_*jk*_ stands for the weight.
Equations (9) and (10) indicate the results of different updated weights.
  (9) $$\begin{array}{c} \Delta W_{jk}\left(n\right)=\frac{\alpha }{1+L}\times \left(\Delta W_{jk}\left(n-1\right)+1\right)\times \delta_{k}\times h_{j}. \end{array}$$
In equation (9),  Δ*W*_*jk*_ stands for the updated weight, *n* expresses the quantity, *α* stands for the learning rate, and *L* points to the total error term. The remaining letters represent the same as in equation (9).
  (10) $$\begin{array}{c} \Delta V_{ij}\left(n\right)=\frac{\alpha }{1+L}\times \left(\Delta V_{ij}\left(n-1\right)+1\right)\times \delta_{k}\times h_{j}. \end{array}$$
In equation (10),  Δ*V*_*ij*_ means another updated weight, and the remaining letters mean the same as in (10).
The threshold values are adjusted concurrently. Equations (11) and (12) present the specific results.
  (11) $$\begin{array}{c} \Delta \theta_{k}\left(n\right)=\frac{\alpha }{1+L}\times \left(\Delta \theta_{k}\left(n-1\right)+1\right)\times \delta_{k}. \end{array}$$
In Equation (11), Δ*θ*_*k*_ means the adjusted threshold value, and the remaining letters express the same as in Equation (10).
  (12) $$\begin{array}{c} \Delta \phi_{j}\left(n\right)=\frac{\alpha }{1+L}\times \left(\Delta \phi_{j}\left(n-1\right)+1\right)\times \delta_{j}. \end{array}$$
In (12),  Δ*ϕ*_*j*_ stands for the adjusted threshold value, and the remaining letters denote the same as in (11).
Finally, the weight and threshold are adjusted uniformly. Equations (13)-(16) display the specific results.
  (13) $$\begin{array}{c} W_{jk}\left(n+1\right)=W_{jk}\left(n\right)+\Delta W_{jk}\left(n\right), \end{array}$$
  (14) $$\begin{array}{c} V_{ij}\left(n+1\right)=V_{ij}\left(n\right)+\Delta V_{ij}\left(n\right), \end{array}$$
  (15) $$\begin{array}{c} \theta_{k}\left(n+1\right)=\theta_{k}\left(n\right)+\Delta \theta_{k}\left(n\right), \end{array}$$
  (16) $$\begin{array}{c} \phi_{j}\left(n+1\right)=\phi_{j}\left(n\right)+\Delta \phi_{j}\left(n\right). \end{array}$$
In equations (13)–(16),  *W*_*jk*_ and *V*_*ij*_ represent different weights, and *θ*_*k*_ and *ϕ*_*j*_ denote different thresholds. The remaining letters represent the same as in equation (12).
The following equation signifies the calculation method of the relationship between output data and input data:
  (17) $$\begin{array}{c} D=\eta \left(\sum_{i=1}^{4}c_{i}d_{i}+a\right). \end{array}$$
In equation (17), *η* represents an activation function, *c*_*i*_ denotes the input information of the neuron, *d*_*i*_ means the weight value corresponding to the neural information element, and *a* stands for the intercept.
The weighted sum of neurons can be obtained according to equation (17), and The following equation shows the specific calculation method.
  (18) $$\begin{array}{c} T_{i}=\sum_{j=1}^{n}u_{ij}a_{j}+c_{j}. \end{array}$$
In equation (18), *T*_*i*_ represents the weighted sum of neurons, *j* represents the neural information element, *u*_*ij*_ means the *i*th weight value corresponding to the neural information element, and *a*_*j*_ indicates the input information corresponding to the neural information element.
Similarly, the activation value of neurons can also be obtained according to equation (18), and the specific calculation method is shown in
  (19) $$\begin{array}{c} f_{i}=\eta \left(T_{i}\right). \end{array}$$
In equation (19), *f*_*i*_ represents the activation value of the *i*th neuron, and the remaining letters represent the same as in the above equations.
The backpropagation algorithm is an important algorithm for neural network training, but a cost function needs to be set before using this algorithm. The following equation reveals the specific calculation method of the cost function.
  (20) $$\begin{array}{c} G\left(b,c\right)=\left[\frac{1}{n}\sum_{i=1}^{n}\left(\frac{1}{2}\left\|\;\right.h_{u,c}{\left(x^{\left(i\right)}-y^{\left(i\right)}\left\|\;\right.\right)}^{2}\right)\right]+\frac{\lambda }{2}. \end{array}$$
In equation (20), *G* means the cost function, *u* denotes the weight value corresponding to the neural information element, *n* refers to the number of layers, *x*^(*i*)^ and *y*^(*i*)^ accord with different training sets, *λ* refers to the random coefficient, *h* stands for the amplitude of the weight, and the remaining letters represent the same as in the above equations. According to equation (20), the gradient descent algorithm can be used to update the network parameters. The following equation displays the specific calculation method:
  (21) $$\begin{array}{c} u_{ij}=b_{ij}-\varepsilon \frac{1}{b_{ij}}G\left(u,c\right). \end{array}$$
In equation (21), the specific meanings of *u*, *G*, and *c* are the same as in the above equations, *i* and *j* represent different neurons, respectively, and *ε* denotes the learning rate.
  (22) $$\begin{array}{c} a_{i}=a_{i}-\varepsilon \frac{1}{c_{i}}G\left(a,c\right). \end{array}$$
In equation (22), *a*_*i*_ represents the intercept corresponding to the *i*th neural information element, and the remaining letters express the same as in the above equations.
Equations (23) and (24) indicate the calculated partial derivatives of (19) and (20).
  (23) $$\begin{array}{c} G\left(u,c\right)=\left[\frac{1}{n}\sum_{i}^{n}G\left(u,c;x^{\left(i\right)},y^{\left(i\right)}\right)\right]+\lambda b_{ij}. \end{array}$$
Letters in equation (23) represent the same as in the above equations.
  (24) $$\begin{array}{c} G\left(a,c\right)=\frac{1}{n}\sum_{i=1}^{n}G\left(a,c;x^{\left(i\right)},y^{\left(i\right)}\right). \end{array}$$
Letters in equation (24) represent the same as in the above equations.
Meanwhile, equation (25) illustrates the calculation method of neuron residual in the output layer.
  (25) $$\begin{array}{c} \gamma_{i}=\frac{1}{2}{\left\|x-h_{u,c}\right\|}^{2}=-\left(x_{i}-e_{i}\right). \end{array}$$
In equation (25), *γ* represents the residual error, *x* refers to the training set, and *e* stands for the input information. The remaining letters express the same meanings as in the above equations.
Equations (26) and (27) show the calculated partial derivatives of equations (21) and (22).
  (26) $$\begin{array}{c} G\left(u,c;x,y\right)=a_{j}\cdot \gamma_{i}. \end{array}$$
Letters in equation (26) represent the same as in the above equations.
  (27) $$\begin{array}{c} G\left(u,c;x,y\right)=\gamma_{i}. \end{array}$$
Letters in equation (27) represent the same as in the above equations.
  (28) $$\begin{array}{c} K_{i}=f\left(C_{i-1}⊙W_{i}+u_{i}\right). \end{array}$$
In equation (28), *K*_*i*_ stands for the characteristic diagram in the *i*th layer of CNN. The symbol ⊙ means the convolution operation between the characteristic diagram in the *i *−* *1th layer and the characteristic diagram in the *i*th layer.
  (29) $$\begin{array}{c} a_{i}=\text{subsampling}\left(a_{i-1}\right). \end{array}$$
Equation (29) signifies the calculation in the pooling layer, and the remaining letters in (29) bespeak the same as in the above equations.
(3) The generating countermeasure network is a DL model and can perform unsupervised learning on complex distribution. The model produces a fairly good output through mutual game learning of at least two modules in the framework, which are the generative model and discriminant model [17]. The model is shown in Figure 5.

Equation (30) indicates the specific calculation method.

(30) $$\begin{array}{c} \min\sum_{m}^{M}L\left(A^{m},B^{m},C^{m}\right)+\ell \text{Reg}\left(C\right). \end{array}$$

In equation (30), *A*^*m*^, *B*^*m*^, *C*^*m*^, respectively, represent the input *A*, *B*, *C* matrix of the *m*th task. *M* stands for the total number of samples, Reg means the regularization constraint, and *ℓ* denotes the weight that controls the regularization constraint.

RETRACTED

The above three models cooperate in the online teaching design of IPE. RNN processes the curriculum language. CNN calculates the specific error and produces the confrontation model. Through discrimination and game, the three can complement and jointly promote the normal operation of IPE.

Visual sensing technology is one of the seven categories of sensing technology. Visual sensors are the direct source of information of the whole machine vision system. It is mainly composed of one or two graphic sensors and is equipped with light projectors and other auxiliary equipment [18]. Vision sensors are used to obtain enough original images to be processed by the machine vision system [19]. The image processing process is shown in Figure 6.

## 3. Research Methods

(1) Interviews on related experts: It means visiting experts in the field of curriculum politics, inviting them to an interview, asking them about the current situation of the development of curriculum politics in China in recent years, and listening to their suggestions and opinions on this aspect, to enhance the science nature and rationality of the paper [20, 21]. (2) Comparative analysis method: It refers to comparing two or more research objects, exploring their similarities and differences, and analyzing, studying, and drawing lessons from good methods. The purpose is to explore the proper online teaching design of curriculum politics [22]. (3) Literature method: It means looking up literature resources. In detail, due to the writing needs of the present work, first, information is queried from online channels such as CNKI, Google Academic, and Wanfang Database; secondly, there are many articles and works from columnists and relevant Internet information; thirdly, many related journals and books are referred in the school library. The collection and summarization of this series of data provide a favorable theoretical basis for the research ideas and methods of this paper [23, 24]. (4) Questionnaire survey method: through setting corresponding questionnaire questions to understand the current situation of online curriculum politics in Chinese courses, the purpose is to reveal the impact of DL and visual sensing technology on curriculum politics [25]. Therefore, 300 questionnaires are randomly distributed to college students in June 2019. To ensure the scientific nature of the questionnaires, discussion on them is made with relevant experts before the questionnaires are distributed. Besides, the unreasonable places are modified. To ensure the corresponding recovery rate, 253 copies are recovered in the form of face-to-face distribution and on-the-spot recovery, with a recovery rate of about 84.3%, and 239 copies are effectively recovered, with an effective recovery rate of 94.5%.

The Kaiser–Meyer–Olkin (KMO) coefficient is introduced to test the data of the questionnaire. Equation (31) specifies the calculation method.

(31) $$\begin{array}{c} KMO=\frac{\sum \sum_{i\neq j}r_{ij}^{2}}{\sum \sum_{i\neq j}r_{ij}^{2}+\sum_{i\neq j}r_{ij}^{2}\cdot 1,2\ldots k}. \end{array}$$

In equation (31), *r* represents the correlation coefficient, *i* denotes the dependent variable, *j* stands for the independent variable, and *k* expresses the quantity.  Table 1 lists the measurement criteria.

RETRACTED

The validity of the data of this questionnaire is analyzed by SPSS 23 with the relevant knowledge of statistics. The *KMO* value is 0.869, ranging from 0.8 to 0.9, and the *p*-value is 0, less than 0.01, which shows that the questionnaire is very suitable for factor analysis, and it has good validity.

## 4. Results

### 4.1. Development Status of Online Curriculum Politics

The questionnaire survey reveals the learning motivation of college students to curriculum politics, as shown in Figure 7.

The values are shown in Table 2.

Figure 7 implies that there are many students interested in curriculum politics, who account for about 85% of the total participants; when it comes to learning objectives, about 60% of students are not very clear or unclear; additionally, about 70% of the students think that curriculum politics are still important; finally, when asked about the course arrangement, 41% of the students think that the class hours are long but scattered. These data can reveal that in most students' ideas, curriculum politics are more than important but necessary to learn. However, there are still problems in the arrangement of class hours and the establishment of learning goals.

The specific results are obtained through the analysis of the students' behavior of learning curriculum politics, as shown in Figure 8.

The values are shown in Table 3.

As Figure 8 suggests, first, students think that from the curriculum politics, what is greatly improved in them are thinking, knowledge, ability, and quality, in order. Besides, what students want to obtain in the ideological and political courses is the cultivation and education of good personal quality, the patriotism education, the cultivation and education of scientific and humanistic quality, and dialectical materialism education, in order. By learning the relevant theories of IPE in class, 35.4% of the students think that they have improved a lot, 32.8% of the students think that there is only some improvement, 19.7% of the students comprehend at least half of the contents, and 12.1% of the students think that there are no differences to them. As the teaching contents taught in class, about 30.8% of the students can often feel them in real life, 41% of them occasionally feel them, 15.5% of them rarely feel them, and 12.7% of them never feel them. Most students want to comprehensively improve themselves through curriculum politics. However, on the one hand, students reckon the knowledge taught in class is disconnected from real life, resulting in that fewer students having strong feelings for the contents. On the other hand, when IPE is carried out mainly focused on theories, teachers make relatively less interaction with students. As for about 31% of the students, they only comprehend a little of the teaching contents.

RETRACTED

### 4.2. Application of DL and Visual Sensing Technology in Curriculum Politics Design

The questionnaire survey shows that there are still some problems in the online teaching design of IPE. In view of this, DL and visual sensing are integrated into the online teaching design of IPE. Now, the semantic segmentation of the image is taken as an example to explore the principle, construction, and training of its segmentation model. The samples are selected from the data sets released on the network and programmed with Python, and TensorFlow is used as the framework. The experiment process is shown in Figure 9.

Figure 9 shows that DL and visual sensing are added to the semantic segmentation of the images of IPE. The research process is divided into four parts: preprocessing the data of IPE, implementing the model, designing the loss function, and training the model. After DL and visual sensing are introduced, the courses before and after the introduction are compared, and the advantages of DL and visual sensing are summarized.

Now, 200 participants are randomly divided into two groups.  Table 4 specifies the experiment results.

A questionnaire survey was conducted in the classroom after adding DL and visual sensing.

A questionnaire survey is conducted on the students after adding DL and visual sensing technology to the curriculum politics.  Figure 10 demonstrates the specific results.

Figure 10 expounds that the average students' concentration time is about 30.4 minutes after DL, and visual sensing technology is introduced into the curriculum politics, while that is only about 29 minutes before the introduction of these two technologies. It implies that the introduction of DL and visual sensing technology into curriculum politics helps to attract students' attention and focus longer. The method is proved to be more conducive to college students' acceptance of curriculum politics.

To test the influence of DL and visual sensing technology on the online teaching of curriculum politics from many aspects, the college students are investigated for their homework submission efficiency after the experiment. Figures 11 and 12 demonstrate the results.

The results are shown in Tables 5 and 6.

Through the comparison of students' homework submission efficiency before and after the experiment, it is found that the change of homework efficiency of gifted students before and after the experiment is not very obvious but tends to be stable. Besides, there is no obvious fluctuation, which shows that the change before and after the experiment still has little impact on the homework submission efficiency of gifted students. The homework submission efficiency of the top students has changed to some extent; especially, the efficiency of the third top student has changed significantly, and his efficiency has been greatly improved to gradually approach that of the top students. It indicates that the impact on the top students has been further improved after the adjustment of teaching contents. Although there is still a gap in the efficiencies of the three middle school students with that of the top students, the fluctuation between them before and after the experiment has gradually narrowed, indicating that the learning attitude of middle school students has been improved compared with that before, which also shows that the adjustment of class strategies has also had a certain positive impact on middle school students.

RETRACTED

Simultaneously, the 200 college students are investigated for their feelings.  Figure 13 displays the results.

Figure 13 illustrates that about 72% of the students like or prefer this mode of class; about 13% of the students do not like this mode; 15% of the students do not always like this mode; about 68% of the students think that this model has improved their learning confidence; about 25% of the students think that their learning confidence has hardly improved; 7% of the students think that it reduces their confidence. In short, adding DL and visual sensing technology helps improve students' enthusiasm in class and confidence in learning, and students' experience increases. A small number of students believe that they have not improved their enthusiasm and learning confidence. The reasons are, on the one hand, they do not have enough acceptor ability; on the other hand, this model needs to be improved in some aspects.

## 5. Conclusions

Through the introduction of DL and visual sensing technology into the online teaching design of curriculum politics, the main conclusions are as follows: (1) after understanding the online teaching of curriculum politics in colleges, it is found that college students have a strong interest in the learning of curriculum politics, and they think it is important, but there are still some situations, such as students' inadequate understanding of the course contents and learning goals; (2) the experimental model is designed to introduce DL and visual sensing technology into the IPE in colleges, which is mainly divided into four parts: data preprocessing, model construction, loss function design, and model training; (3) by integrating DL and visual sensing technology into the IPE in colleges, it is found that students' concentration time in class becomes longer, the classroom atmosphere becomes more active, and students' homework submission efficiency becomes higher. Simultaneously, most students also have more confidence in their own and are more active in learning. The conclusion is that DL and visual sensing technology can optimize the teaching design of curriculum politics.

RETRACTED

Due to the limited energy, the present work has some limitations in data acquisition, resulting in some deviations in the inspection of relevant data. Besides, there is no discussion on the economic investment of DL and visual sensing technology in the process of online curriculum politics. In the follow-up, the benefit can be evaluated according to the specific situation, so that suggestions and opinions can better optimize the problems existing in the curriculum politics.

## Figures and Tables

**Figure 1:** Theoretical basis of curriculum politics.

**Figure 2:** DL model.

**Figure 3:** Recurrent neural network.

**Figure 4:** Convolutional neural network.

**Figure 5:** The model of the GAN.

**Figure 6:** Image processing process.

**Figure 7:** The learning motivation of college students to the curriculum politics ((a) the students' interest in the curriculum politics; (b) the students' clarity of the goals of the curriculum politics; (c) the students' attention to the curriculum politics; (d) the class arrangement of the curriculum politics).

**Figure 8:** Analysis of college students' learning behavior in the curriculum politics ((a) the degree of students' improvement from curriculum politics; (b) the elements students expect to learn from curriculum politics; (c) students' cognition of curriculum politics; (d) the correlation between curriculum politics and real-life).

**Figure 9:** Application of DL and visual sensing in IPE.

**Figure 10:** Students' concentration time of different types of courses.

**Figure 11:** Students' homework submission efficiency in the early stage of the experiment.

**Figure 12:** Submission efficiency of students' homework in the later stage of the experiment.

**Figure 13:** Evaluation of students' feelings after introducing DL and visual sensing technology.

**Table 1:** Measurement criteria of the *KMO*.

Type	Range of values	Factor analysis is appropriate
*KMO* value	*KMO* < 0.9	Very much suitable
	0.8 <*KMO*≤ 0.9	Very suitable
	0.7 <*KMO*≤ 0.8	Fit
	0.6 <*KMO*≤ 0.7	Not very suitable
	0.5 <*KMO*≤ 0.6	Barely fit
	*KMO*≤ 0.5	Unsuited

**Table 2:** College students' motivation for IPE.

Type	Motivational situation	Number of people	Proportion
Degree of interest	Particularly interested	50	21.1%
	More interested	105	43.9%
	Generally interested	50	21.1%
	Very uninterested	34	13.9%

Clarity of learning objectives	Very clear	37	15.5
	Relatively clear	64	26.6
	It's a little fuzzy	81	34
	Vague	57	23.9

Emphasis on ideological and political education	Unimportance	23	9.7
	Not very important	45	18.7
	More important	114	47.7
	Very important	57	23.9

Class arrangement	Many and concentrated classes	51	21.4
	More class hours but scattered	98	41
	More class hours but scattered	59	24.7
	Few and scattered classes	31	12.9

RETRACTED

**Table 3:** College students' behavior in the learning process of IPE.

Type	Motivational situation	Number of people	Proportion
Student promotion	Knowledge	169	70.6
	Thinking	182	76.3
	Ability	165	68.8
	Quality	146	61.2

Elements learned	Dialectical materialism	168	70.2
	Patriotism education	182	76.3
	Cultivation of humanistic quality	174	72.6
	Personal quality training	193	80.7

Course ideological and political cognition	Improve a lot	85	35.4
	Improve some	78	32.8
	Half knowledge and half solution	47	19.7
	No change	30	12.1

Relevance to real life	Always in touch	74	30.8
	Often feel	98	41
	Rarely felt	37	15.5
	Never felt it	30	12.7

**Table 4:** Number and proportion of college students.

Group	People number	Proportion (%)
Group one	100	50
Group two	100	50

**Table 5:** Submission efficiency of students' homework in the early stage of the experiment.

Type frequency	Secondary students 1	Secondary students 2	Secondary students 3	Top student 1	Top student 2	Top student 3	Gifted students 1	Gifted students 2	Gifted students 3
0.5	0.85717	1.0677	1.18598	2.30445	2.5679	2.34389	3.38371	3.52799	3.60719
1.5	0.63669	1.17628	0.89958	2.75511	2.57083	2.36038	3.39996	3.47858	3.71549
2.5	0.7455	1.3374	0.96902	2.54801	2.37686	2.49492	3.12659	3.48201	3.87667
3.5	0.86676	1.36685	1.27491	2.41943	2.7089	2.53792	3.39356	3.63007	3.72198
4.5	0.85716	0.75183	1.01511	2.63354	2.75163	2.7119	3.54139	3.3438	3.80438
5.5	0.50519	0.61042	0.80779	2.75496	2.80762	2.57082	3.33403	3.53149	3.66294
6.5	0.81111	0.94276	0.98226	2.81118	2.5873	2.9294	3.69245	3.7584	3.7713
7.5	1.01174	1.09065	0.84059	2.91954	2.52477	2.72201	3.40621	3.38015	3.73557

**Table 6:** Submission efficiency of students' homework in the later stage of the experiment.

Type frequency	Secondary students 1	Secondary students 2	Secondary students 3	Top student 1	Top student 2	Top student 3	Gifted students 1	Gifted students 2
8.5	0.41449	0.96616	1.04656	2.36846	2.54092	2.72478	3.44894	3.50526
9.5	0.78337	0.78351	0.82933	2.63406	2.62252	2.77184	3.37999	3.67875
10.5	0.96839	0.88796	1.08337	2.46275	2.78458	3.01442	3.51908	3.77184
11.5	0.9695	0.75116	1.05003	2.63621	2.82024	2.96951	3.45102	3.72683
12.5	0.91293	1.01676	1.07416	2.9018	2.8673	3.05145	3.36042	3.7283
13.5	0.86735	0.88002	1.14423	2.59267	2.77662	3.14447	3.45355	3.54559
14.5	0.69604	1.15709	1.20292	2.82369	2.94997	3.13385	3.40851	3.81218
15.5	0.88127	1.08925	1.20414	2.76729	2.87091	3.03172	3.57078	3.54908
16.5	0.96275	0.94093	0.98681	2.55009	2.84891	3.00986	3.34218	3.59607
17.5	0.83757	0.99959	1.24092	2.76962	2.85009	3.04556	3.44667	3.6891

RETRACTED

## Data Availability

The data used to support the findings of this study are available from the corresponding author upon request.

## References

[1] Lee J. (2020). Integration of digital twin and deep learning in cyber-physical systems: towards smart manufacturing. *Sustainability*.

[2] Qiu Z. (2017). Deep learning and its applications to machine health monitoring. Mechanical Systems and Signal Processing. *IEEE Syst J*.

[3] Zhu Z. (2019). State of the art: secure mobile payment. *IEEE Access*.

[4] Shi J. (2018). Emv-compatible offline mobile payment protocol with mutual authentication. *Sensors*.

[5] Mandalorian Z. (2018). Why do people switch mobile payment service platforms? an empirical study in Taiwan. *Technology in Society*.

[6] Saussure F. A. (2018). Application of optical remote sensing in rubber plantations: a systematic review. *Remote Sensing*.

[7] Tissters L. (2019). Will users keep using mobile payment? it depends on trust and cognitive perspectives. *Procedia Computer Science*.

[8] Hsiao M. (2020). Mobile payment services as a facilitator of value co-creation: a conceptual framework. Journal of High Technology Management Research. *Science Observation*.

[9] Liao L. (2020). Mobile payment and online to offline retail business models. Journal of Retailing and Consumer Services. *Popular Science and Technology*.

[10] Gong X. (2020). Transition from web to mobile payment services: the triple effects of status quo inertia. International Journal of Information Management. *Journal of Image and Graphics*.

[11] Wang Y. (2020). Mobile payment and informal business: evidence from China’s household panel data. *Progress in Laser and Optoelectronics*.

[12] Vincent O. (2020). An identity-based elliptic curve cryptography for mobile payment security. *Computer Science*.

[13] Jia D. (2018). Influence of habits on mobile payment acceptance: an ecosystem perspective. *Information Systems Frontiers*.

[14] Esfahani B. (2021). The influence of individual differences on nfc-based mobile payment adoption in restaurant industry. *Ieee Journal of Selected Topics in Applied Earth Observations and Remote Sensing*.

[15] Verma S. (2020). The effect of government regulations on continuance intention of in-store proximity mobile payment services. *International Journal of Bank Marketing*.

RETRACTED

[16] Nelloh W. (2021). Will users keep using mobile payment? it depends on trust and cognitive perspectives. *Procedia Computer Science*.

[17] Bojjagani N. (2021). A secure end-to-end proximity nfc-based mobile payment protocol. *Xiehe Medical Journal*.

[18] Chalee K. (2020). A lightweight and secure nfc‐base mobile payment protocol ensuring fair exchange based on a hybrid encryption algorithm with formal verification. International Journal of Communication Systems. *Economic Management Digest*.

[19] Zhang M. (2021). Spillover effects from web to mobile payment services: the role of relevant schema and schematic fit. *Internet Research*.

[20] Khn I. (2021). Mobile payment - eine vertrauensfrage. *Textil Wirtschaft*.

[21] Deng M. (2020). The specific application of microelectronic control electromechanical equipment in industry. *Electronics World*.

[22] Wang C., Fan J. H., Lin S. M. (2020). Research on the correlation between optical remote sensing vegetation index and sar remote sensing parameters and its main influencing factors. *Remote sensing of land and resources*.

[23] Karsen M. (2021). Technological factors of mobile payment: a systematic literature review. *Procedia Computer Science*.

[24] Sinha N. (2020). Assessment of mobile technology use in the emerging market: analyzing intention to use m-payment services in India. *Telecommunications Policy*.

[25] Bojjagani S. (2020). Systematic survey of mobile payments, protocols, and security infrastructure. *Journal of Ambient Intelligence and Humanized Computing*.

